The article "Prediction and Elucidation of Triglycerides Levels Using a Machine Learning and Linear Fuzzy Modelling Approach" was published in 2022. Journal: Biomed Res Int.

# Prediction and Elucidation of Triglycerides Levels Using a Machine Learning and Linear Fuzzy Modelling Approach

**DOI:** 10.1155/2022/7511806

**Published:** 2022-02-24

**Authors:** Wan Muhamad Amir W Ahmad, Faraz Ahmed, Nor Farid Mohd Noor, Nor Azlida Aleng, Farah Muna Mohamad Ghazali, Mohammad Khursheed Alam

**Affiliations:** ^1^School of Dental Sciences, Health Campus, Universiti Sains Malaysia (USM), 16150 Kubang Kerian, Kota Bharu, Kelantan, Malaysia; ^2^Faculty of Medicine, Universiti Sultan Zainal Abidin (UniSZA), Medical Campus, Jalan Sultan Mahmud, 20400 Kuala Terengganu, Terengganu Darul Iman, Malaysia; ^3^Faculty of Ocean Engineering Technology and Informatics, Universiti Malaysia Terengganu (UMT), 21030 Kuala Nerus, Terengganu, Malaysia; ^4^Preventive Dentistry Department, College of Dentistry, Jouf University, Sakaka 72345, Saudi Arabia; ^5^Center for Transdisciplinary Research (CFTR), Saveetha Dental College, Saveetha Institute of Medical and Technical Sciences, Saveetha University, Chennai, India; ^6^Department of Public Health, Faculty of Allied Health Sciences, Daffodil lnternational University, Dhaka, Bangladesh

## Abstract

**Introduction:**

Triglycerides are lipids composed of fatty acids that provide energy to the cell. These compounds are delivered to the body's cells via lipoproteins found in the bloodstream. Increased blood triglyceride levels have been associated with high-fat or high-carbohydrate diets. Generally, increased triglyceride levels occur in conjunction with other symptoms that are difficult to notice and recognize.

**Objectives:**

The study's goal was to develop and predict the model that could be used to explain the relationship between triglycerides and waist circumference, high-density lipoprotein (HDL), and hypertension status by determining the relationship between triglycerides and waist circumference, HDL, and hypertension status. This model was developed using qualitative predictor variables and incorporated data bootstrapping multilayer perceptron neural networks and fuzzy linear regression. *Materials and procedures*. This was a public health study that combined retrospective data analysis with methodology development. The medical records of patients who attended outpatient clinics at Hospital Universiti Sains Malaysia (USM) were collected and analyzed. This was to provide a more extensive illustration of the methods developed. Screening and selection of patient data were necessary following the inclusion and exclusion criteria. The patient's medical record was used to obtain triglycerides, high-density lipoprotein (HDL), waist circumference, and hypertension status. Due to the critical nature of the variable, it was chosen to aid the clinical expert. The R-Studio software was used to develop the associated syntax for the hybrid model, which would define the association between the examined variables. The purpose of this study is to create a technique for the clinical trial design that utilizes bootstrapping, Qualitative Predictor Variables (QPV), Multiple Linear Regression (MLR), Artificial Neural Networks (ANNs), and Fuzzy Regression (FR). All analyses were performed using the newly introduced R syntax. The research developed a fuzzy linear model that increased modelling performance by incorporating clinically significant factors and validated variables via Multilayer Perceptron (MLP).

The article "Prediction and Elucidation of Triglycerides Levels Using a Machine Learning and Linear Fuzzy Modelling Approach" was published in 2022. Journal: Biomed Res Int.

**Conclusion:**

The proposed technique for modelling and prediction appeared to be the ideal combination of bootstrap, Multilayer Feed Forward (MLFF) neural network, and fuzzy linear regression. The created syntax is currently being evaluated and validated clinically. For modelling and prediction, the proposed technique looked to be the best, as it incorporated bootstrap, MLFF neural network, and fuzzy linear regression. The established syntax is now being utilized in the clinic to evaluate and validate the outcome. In terms of variable selection, modelling, and model validation, this strategy was superior to earlier approaches for fuzzy regression modelling.

## 1. Introduction

Triglycerides are fat-soluble fatty acids that circulate throughout the body. Triglycerides account for most of the fats we ingest, including butter, margarine, and oils. Excess calories, alcohol, and sugar are converted to triglycerides deposited in the body's fat cells. Triglycerides can be assessed fasting or nonfasting, with levels between 2 and 10 mmol/L indicating an elevated risk of cardiovascular disease and levels greater than ten mmol/L indicating an increased risk of acute pancreatitis and possibly cardiovascular disease. Elevated triglyceride levels are significantly related to low HDL cholesterol levels. Elevated triglyceride levels are frequently connected with other heart disease and stroke risk factors, such as obesity and metabolic syndrome. A prior study connected higher waist circumference with increased systolic and diastolic blood pressures, hyperglycemia, HDL cholesterol, and triglycerides [1, 2]. Obesity and uncontrolled diabetes are the two most common causes of elevated triglycerides. Triglycerides can increase if someone is overweight and inactive, especially if they consume a lot of carbs or sugary meals or consume a lot of alcohol. Apart from that, obesity and poorly controlled diabetes are the two most common causes of high triglycerides. Triglycerides can be raised if someone is overweight and inactive, especially if they consume a lot of carbs or sugary meals or if they drink alcohol. Minimum test concentrations should be 150 mg/dL (1.69 mmol/L). The borderline is considered to be elevated, with values ranging from 150 mg/dL (1.69 mmol/L) to 199 mg/dL (2.25 mmol/L) being considered high. The levels are considered to be high between 200 and 499 mg/dL (2,26-5,63 mmol/L). Levels exceeding 500 mg/dL are extremely high (5.64 mmol/L) [1, 3, 4]. This article is significant for several reasons, most significantly for modelling and inference. The essay highlights the inherent limitations of most of the components of a developing hybrid model that integrates linear regression, data bootstrapping, neural networks, and a qualitative predictor variable. The second contribution of this study is unique in that it proves the utility of the bootstrap, multiple linear regression, and multilayer perceptron in self-control theory literature. This information would be highly beneficial in terms of triglyceride management. Additionally, this study intends to provide helpful information and a better knowledge of triglycerides concerning the variables chosen, which included waist circumference, high-density lipoprotein, and blood pressure parameters. This effort will increase our understanding of triglyceride modelling's mechanical behaviour, particularly methodological advancement. [5–9]. The main purpose was to develop and predict the model which determines these relationships effectively and significantly.

The article "Prediction and Elucidation of Triglycerides Levels Using a Machine Learning and Linear Fuzzy Modelling Approach" was published in 2022. Journal: Biomed Res Int.

## 2. Materials and Methods

### 2.1. Data Collection

This study assessed data from patients who visited the Hospital Universiti Sains Malaysia's outpatient clinic (USM). This study enrolled a total of 14 patients. The data description for the study's selected variables is summarized in Table 1.

### 2.2. Study Design

A methodology based on the design of a computational retrospective study. The study case was illustrated by Triglycerides (Y), Waist (X_1_), High-Density Lipoprotein (X_2_), and Hypertension status (X_3_). In fuzzy linear regression, the qualitative predictor variable, also known as dummy variables, is used as an independent variable. Before using this procedure, a dummy variable must be created before conducting the analysis. This necessitated using a set of dummy variables that was one less than the total number of categories. A dummy variable is a categorical variable with values 0 and 1 used to compare various types. A number of 1 indicate that the case falls into a particular category, whereas a value of 0 indicates that it does not. It is a nonsignificant dummy variable. The Universiti Sains Malaysia Research Ethics and Committee (Human) (USM/JEPeM/17040225) approved the study. The patient's privacy and medical condition are both protected.

The article "Prediction and Elucidation of Triglycerides Levels Using a Machine Learning and Linear Fuzzy Modelling Approach" was published in 2022. Journal: Biomed Res Int.

### 2.3. Modelling of Computational Biometry

The data were evaluated for links to triglyceride levels. The data were examined using the R-Studio software and the syntax that was implemented. The advanced strategy in this methodology is a combined model that employs the bootstrap, multilayer perceptron (MLP), and multiple linear regression (MLR) techniques. The Multilayer Perceptron (MLP) is a type of feedforward artificial neural network that is frequently used. MLP is a three-layer architecture consisting of an input layer, a hidden layer, and an output layer [4, 9–11].

### 2.4. Regression with Qualitative Predictor Variable

Qualitative predictor variables with a class are represented by *a*-1 indicator variables with the values 0 and 1. Dummy variables or binary variables are common names for indicator variables. If a qualitative variable has more than two classes, the regression model will include additional indicator variables. Let us say we have (*Y*), (*X*_1_ = Waist), (*X*_2_ = HDL), and (*X*_3_ = Hypertension)

(1) $$\begin{array}{c} \text{Triglycerides}=\beta_{0}+\beta_{1}\text{Waist}+\beta_{2}\text{ HDL}+\beta_{3}\text{ Hypertension}+\varepsilon , \end{array}$$

where Hypertension is a variable with three classes: normal, borderline, and hypertension. Therefore, it needs two indicators. Let us define the variable as follows:

(2) $$\begin{array}{c} \text{Borderline}=\left\{\begin{array}{cc} 0 & \text{No}\\ 1 & \text{Yes} \end{array}\right.\text{and High Blood Pressure}=\left\{\begin{array}{cc} 0 & \text{No}\\ 1 & \text{Yes} \end{array}\right. \end{array}$$

### 2.5. Bootstrap

Bootstrap begins by randomly selecting a sample of the population and then computing sample statistics. After several replications of the initial samples, the bootstrap generates a pseudopopulation by using several substitution samples. After several repetitions of the initial samples, the bootstrap generates a pseudopopulation by using several substitution samples. With substitution, random sampling produces samples that are not identical to the original sample. The bootstrap calculates statistics for each sample as it draws the sample with replacement [6, 7].

### 2.6. Multilayer Perceptron (MLP)

The multilayer perceptron is the most frequently used type of artificial neural network [9, 10]. MLP is composed of three layers: the input, the hidden, and the output. Because this analysis contains only one dependent variable, the output node is unique within the research sample. The strength of this model is to lead the machine learning algorithm also can be used for complex nonlinear problems and can be achieved even with smaller data. Equation $\hat{Y}=g_{i}\left(\sum_{j=1}^{2}n_{j}+E_{2}\right)\;i=1,2;$ constructs an MLP with N input nodes, H hidden nodes, and a single output node. The MLP with N input nodes, H hidden nodes, and a single output node is shown in Figure 1.

The article "Prediction and Elucidation of Triglycerides Levels Using a Machine Learning and Linear Fuzzy Modelling Approach" was published in 2022. Journal: Biomed Res Int.

The value $\hat{Y}$ is given as $\hat{Y}=g_{2}\left(\sum_{j=1}^{2}n_{j}+E_{2}\right)$, where *E*_2_ is the bias for the output node and *g* is an activation function. The value of a hidden node *n*_*j*_ is given as *n*_*j*_ = *g*_*i*_(∑_*j*=1_^2^*v*_*ji*_*x*_*i*_ + *E*_1_)_,_ where *E*_1_ is the bias for the output node and *g* is an activation function, where *v*_*ji*_ the output *weight* from input node *i* to hidden node *j,E*_1_ is the bias for hidden node *j* where *j* = 1, 2 and *x_i_* are the independent variables. The MLP's general architecture is represented in Figure 1. The MLP procedure for the variable selection will be used as the input for the multiple logistic regression [1, 3, 4, 9].

### 2.7. Fuzzy Regression Model Using Possibilistic

Regression analysis is a statistical technique for determining the relationship between variables with a cause and effect relationship. A multilinear regression model contains only one dependent variable and an infinite number of independent variables [4]. Multivariate regression analysis attempts to account for the variation in independent variables that occurs concurrently with the variation in the dependent variable. This section uses a fuzzy regression model to deduce the underlying relationship between triglycerides and the selected explanatory variables. A fuzzy regression model is used in a fuzzy environment to determine the functional relationship between dependent and independent variables. A fuzzy regression model can be written as *Y* = *Z*_0_ + *Z*_1_ *x*_1_ + *Z*_2_ *x*_2_ + ⋯+*Z*_*k*_ *x*_*k*_; here, the explanation variables *x*_*i*_′*s* are assumed to be precise. However, the equation above indicates that the response variable *Y* is not discrete but rather fuzzy, which applies to the parameters. Our objective is to estimate these parameters. In the following discussion, assume that symmetric fuzzy numbers are capable of being expressed as intervals. Their models adopted the general form proposed by Tanaka et al. (1982). The model is as follows:

(3) $$\begin{array}{c} {\tilde{Y}}_{i}={\tilde{A}}_{0}+{\tilde{A}}_{1}x_{1}+\cdots +{\tilde{A}}_{n}x_{n}\text{ or}{\tilde{Y}}_{i}={\tilde{A}}_{0}+\overset{n}{\underset{i=1}{\sum }}{\tilde{A}}_{i}x_{i}, \end{array}$$

where $\tilde{Y}$ is the fuzzy output, output ${\tilde{A}}_{i}$, j =1,2,…, *n*. is a fuzzy coefficient (Figure 2), and (*x = x_1_, x_2_,…, x_n_*) is a dimension non-fuzzy input vector. The fuzzy component was assumed to be a triangle (TFNs) (Figure 3).

The article "Prediction and Elucidation of Triglycerides Levels Using a Machine Learning and Linear Fuzzy Modelling Approach" was published in 2022. Journal: Biomed Res Int.

Defining the parameter as

(4) $$\begin{array}{c} {\tilde{A}}_{j}=\left\{a_{j},c_{j}\right\}=\left\{{\tilde{A}}_{j}:{\text{a}}_{\text{j}}-\text{cj}\leq {\tilde{A}}_{j}\leq a_{j}+c_{j}\right\}j=0,1,\cdots ,n \end{array}$$

and restricting consideration to the case where only the coefficient are fuzzy, we can write

(5) $$\begin{array}{c} {\tilde{Y}}_{i}={\tilde{A}}_{0}+\overset{n}{\underset{i=1}{\sum }}{\tilde{A}}_{i}x_{ij}=\left(a_{0},c_{0}\right)+\overset{n}{\underset{j=1}{\sum }}\left(a_{j},c_{j}\right)x_{ij}. \end{array}$$

This is a beneficial formulation because it explicitly portrays the mode of the spreads of the fuzzy parameters. In a subsequent section, we explore fuzzy independent variables.

In this case, the proposed fuzzy model is given as follows:

(6) $$\begin{array}{c} \text{Triglycerides}={\tilde{A}}_{1}\;\text{Waist}+{\tilde{A}}_{2}\;\text{Hdl}+{\tilde{A}}_{3}\;\text{Borderline}+{\tilde{A}}_{4}\;\text{Hypertension},\\ \text{Triglycerides}=\left\{a_{1},c_{1}\right\}\text{Waist}+\left\{a_{2},c_{2}\right\}\text{Hdl}+\left\{a_{3},c_{3}\right\}\text{Borderline}+\left\{a_{4},c_{4}\right\}\text{Hypertension}. \end{array}$$

The result for the model is displayed in Table 2. The fuzzy regression is fitting through the R Software. The full step by step method is given as follows (Figure 4):

Figure 4 illustrates the entire procedure for developing the statistical model. The clinical expert selects the variables to be used before beginning the data collection process. The study's strength is that it looks at a model that takes clinically relevant variables into account. Special consideration should be given to the data for the qualitative predictor variable (see section Qualitative Predictor Variable). Additional analysis is performed using the bootstrap procedure. The bootstrap procedure creates a sample of the same size as the original sample, but each observation is repeated multiple times and omitted. Data preparation will be followed by the construction of a multilayer perceptron neural network (MLPNN), a linear model (LM), and a fuzzy regression (FR) model. The entire procedure for developing the statistical model is depicted in Figure 4. The clinical expert determines the variables to be used before initiating the data collection process. The study's strength is that it examines a model with clinically significant variables. Special consideration must be given to the data for the qualitative predictor variable (see section Qualitative Predictor Variable). The bootstrap procedure is used to conduct additional analysis. The bootstrap procedure generates a sample of the same size as the original sample, but with each observation included multiple times and others omitted [6, 7].

The article "Prediction and Elucidation of Triglycerides Levels Using a Machine Learning and Linear Fuzzy Modelling Approach" was published in 2022. Journal: Biomed Res Int.

## 3. Results

Developing a model that could be used to explain the relationship between triglycerides and waist circumference, high-density lipoprotein (HDL), and hypertension status was the study's goal. This was accomplished by determining the relationship between triglycerides, waist circumference (and thus HDL), and hypertension. In this section, the obtained result will be divided into three different phases.

### 3.1. Phase I: Result for Modelling Multilayer Perceptron (MLP) with One Hidden Layer Approach

The architecture of the MLP is represented in Figure 5, with four input nodes, one hidden layer, and one output node. The variable validation was determined in this section using the developed MLP methodology. The most appropriate model for the case is one hidden layer of MLP. There are three selected variables in this case: Waist, HDL, and Blood Pressure Status. The triglycerides level has been significantly influenced by four factors: waist circumference, high-density lipoprotein, and blood pressure reading status. Blood pressure status is a categorical data set divided into normal, borderline, and high. This study aims at investigating the performance of an MLP neural network with MLR and fuzzy regression. The best model for MLP will be a combination of selected variables that produces a low mean squared error NN (MSE-forecasts the network) to measure how far the predictions deviate from the real data. MSE.net has a value of 0.586234 in this case. The output node is set to a single value, Triglycerides (a dependent variable) in this study. The train to test split is 70 : 30; 90% of the data is available for network training and the remaining 10% for network testing.

### 3.2. Phase II: Result for Multiple Linear Regression

The results of the multiple regression modelling are summarized in Table 2. The model is shown below.

(7) $$\begin{array}{c} \text{Triglycerides}=79.43008+0.33490\text{Waist}+0.57861\text{HDL}+8.55657\text{Border}+19.93486\text{Hyper}. \end{array}$$

The Waist reading (*β*_1_ = 79.43008; *p* < 0.05), HDL (*β*_2_ = 0.33490; *p* < 0.05), borderline reading (*β*_3_ = 0.57861; *p* < 0.05), and Hypertension (*β*_4_ = 8.55657; p < 0.05) show a significant relationship toward the triglycerides. However, the *r*-squared value of 0.8629 (86%) indicated the greater fit of the model to predict a trend.

### 3.3. Phase III: Result for the Fuzzy regression

This paper provides only a fuzzy regression modelling associated with the relationship triglycerides. The primary purpose of this paper is to demonstrate possible techniques that can be employed to explain such relationships. Below is the obtained result of the fuzzy regression.

The article "Prediction and Elucidation of Triglycerides Levels Using a Machine Learning and Linear Fuzzy Modelling Approach" was published in 2022. Journal: Biomed Res Int.

Table 3 shows the result of fuzzy linear regression. Therefore, the fuzzy regression model corresponding to the result can be written as follows.

The central tendency of the fuzzy regression model:

(8) $$\begin{array}{c} \text{Trig}=74.4777+0.4173*\text{Waist}+0.5386*\text{Hdl}+7.4337*\text{Bord}+18.6991*\text{Hyper}. \end{array}$$

Lower boundary of the model support interval:

(9) $$\begin{array}{c} \text{Trig}=72.0179+0.4173*\text{Waist}+0.5386*\text{Hdl}+7.4337*\text{Bord}+12.2426*\text{Hyper}. \end{array}$$

Upper boundary of the model support interval:

(10) $$\begin{array}{c} \text{Trig}=76.9333+0.4173*\text{Waist}+0.5386*\text{Hdl}+7.4337*\text{Bord}+34.7371*\text{Hyper}. \end{array}$$

Fuzzy regression based on the model using possibilistic is being proposed. Equation (8), Equation (9), and Equation (10) give the fuzzy regression model according to the central tendency of the fuzzy regression model, the lower boundary of the model support interval, and upper boundary of the model support interval. According to the findings, the Waist, high-density lipoprotein (HDL), borderline, or hypertension contribute to triglyceride levels. It has been positively associated with triglyceride levels. All the variables were validated through the MLP neural network, and Mean Squared Error NN (MSE-Network Projection) is 0.02377. The smallest MSE of the neural network model shows the best variable selection combination in the model. It can be shown that the hypertension factor gives the most significant influence to the level of lipoprotein (HDL), borderline, or hypertension status, contributing to triglycerides.

## 4. Discussion and Conclusion

Triglycerides are a type of lipid that stores and transports energy. Serum TG is derived from two sources: intestinal absorption and liver synthesis. They are the most common type of fat digested in the body, and they can either be consumed or produced [2]. The goal of this research is to show that triglycerides and circumference have a relationship. Edwina et al. published a study in 2018 in which they measured the waist circumference of 30 people with high triglycerides during their visit. According to the study, there is a strong correlation between triglyceride levels and waist circumference [12]. Our model suggested HDL was directly associated with the increase of triglycerides; however, this result was contradicted with one study which suggested that increased triglyceride levels are associated with decreased HDL cholesterol levels [13], which is associated with an increased risk of ischemic heart disease (IHD). Increased triglyceride levels in the presence of elevated LDL (bad) cholesterol or low HDL (good) cholesterol have been linked to fatty accumulation within the artery walls, increasing the risk of heart attack and stroke. The level of HDL cholesterol is inversely related to the level of triglycerides in the blood. In hypertriglyceridemic patients, HDL particles are more enriched in triglycerides than normal HDL particles. This is because the cholesterol ester in the lipoprotein core of the HDL particle is replaced with triglycerides. Additionally, triglyceride-enriched HDL is more efficiently catabolized. Additionally, researchers discovered a link between high-density lipoprotein (HDL) cholesterol and triglycerides. As a general rule, divide the triglyceride level by the HDL “good” cholesterol level. The ratio of triglycerides to HDL “good” cholesterol should be less than 2, four is considered normal, and six is excessive. In this case, a lower ratio is preferable. As triglyceride levels fall and HDL levels rise, the ratio decreases. [1, 3, 10]. The primary goals were to develop, validate, and test a regression modelling methodology. The primary objective of this project was to develop and implement techniques in the field of medical statistics by combining the bootstrapping procedure with artificial neural networks to validate variable selection and linear modelling to complete the modelling process. Clinical expert opinion is included in the variable selection process. At the start of the operation, the bootstrap method generates a mega file from the original data set. The bootstrap procedure, on the other hand, generates a massive file replacement sample. Thirdly, the bootstrap method calculates and saves sample statistics. Fourthly, the bootstrap method iteratively repeats this process, sometimes thousands of times. At the fifth stage, the data is prepared for the next procedure. The R syntax algorithm enables the application to be integrated with the methodology concept. The first step is to select variables in consultation with a professional. The bootstrap will then be applied to the selected data. Training and testing data will be separated. The R syntax algorithm connects the application to the concept of method-based methodology. The first step, with the assistance of a medical expert, is to select variables. Following that, the data will be subjected to the bootstrap procedure. At this point, 70% of the bootstrap data will be designated as a training dataset and 30% as a testing dataset. The training dataset will be used to construct the model, while the validation dataset will be used to verify it. The Waist, HDL, and blood pressure status all have a significant effect on triglycerides, according to a multilayer perceptron analysis, and these results are in line with the recent study done on elderly Japanese men [14], concluding that triglycerides are positively associated with blood pressure and with hypertension [15].

The article "Prediction and Elucidation of Triglycerides Levels Using a Machine Learning and Linear Fuzzy Modelling Approach" was published in 2022. Journal: Biomed Res Int.

The average square error derived from the multilayer perceptron analysis can be seen. This value was determined after taking into account the training and test sets. It is preferable to obtain a result with the lowest PMSE value. As a result, the study was successful, and the decision-maker received the best possible results. Due to the incorporation of statistical formulations, computation using the developed R syntax, and the neural net package, the proposed methodology resulted in highly successful ANNs. The R neural net package includes the necessary components for building artificial neural networks (ANNs) with various hidden layers and neurons. The most difficult tasks are selecting appropriate input parameters, preparing data, and standardizing it for ANN.

The purpose of this article is to develop a hybrid method that incorporates bootstrapping, quality predictor variables, multilayer perceptron analysis, and multiple linear regression. The R syntax for this methodology was designed to ensure that the researcher fully understood the illustration. In this study, triglycerides were the dependent variable, while waist circumference, HDL, and blood pressure were the independent variables. As a result of the developed model, factors emerged as the most significant factors. When performing multiple linear regressions, the rule of qualitative predictor variables must be followed. In our study, the hybrid model demonstrates that this significant conclusion enables us to understand better the hybrid method's utility and relative contribution to the outcome. This discovery has the most significant potential for further statistical modelling for educational purposes and the decision-maker among the stakeholders.

The proposed strategy and the acquired results demonstrate the superiority of the hybrid model technique given in this work.

## Figures and Tables

**Figure 1:** Two hidden layers, N input nodes, H hidden nodes, and one output node make up the basic MLP architecture.

**Figure 2:** Fuzzy coefficient.

**Figure 3:** Symmetrical fuzzy parameter.

**Figure 4:** The flowchart of the proposed statistical modelling.

**Figure 5:** The result of MLP architecture and multiple linear regression. MLP comprises one hidden layer, N input nodes, H hidden nodes, and one output node.

The article "Prediction and Elucidation of Triglycerides Levels Using a Machine Learning and Linear Fuzzy Modelling Approach" was published in 2022. Journal: Biomed Res Int.

**Table 1:** Data Description of the selected blood profile.

Variable	Code	Description
Trig	Y	Triglyceride levels are measured
Waist_read	X1	Waist circumference is measured
HDL_read	X2	High-density lipoprotein (HDL) is measured
Hypertension_read	X3	0 = Normal blood pressure 1 = borderline 2 = high blood pressure

**Table 2:** Result of multiple linear regression with combining the bootstrap method.

Variable	Estimate	Std error	*t*-value	*P*-value
Intercept	79.43008	2.63104	30.19	<0.01
Waist	0.33490	0.02812	11.91	<0.01
HDL	0.57861	0.02086	27.74	<0.01
Border	8.55657	0.71685	11.94	<0.01
Hyper	19.93486	0.75571	26.38	<0.01

Multiple Linear Regression was applied.

**Table 3:** Result of fuzzy linear regression with combining the bootstrap method.

	Central tendency	Lower boundary	Upper boundary
(Intercept)	74.4777	72.01789	76.93323
Waist	0.41729	0.41729	0.41729
Hdl	0.53860	0.53859	0.53859
Bord	7.43368	7.43368	7.43368
Hyper	18.69911	12.24262	34.73710

## Data Availability

All data are available within the manuscript.
